The article "Prognosis and Therapeutic Efficacy Prediction of Adrenocortical Carcinoma Based on a Necroptosis-Associated Gene Signature" was retracted in 2024. Reasons: signs of a paper mill; suspected computer-generated content; unreliable results or conclusions; concerns about the data.

# Prognosis and Therapeutic Efficacy Prediction of Adrenocortical Carcinoma Based on a Necroptosis-Associated Gene Signature

**DOI:** 10.1155/2022/8740408

**Published:** 2022-05-19

**Authors:** Dan Ji, Rongfang Zhong, Song Fan

**Affiliations:** ^1^Department of Basic Medicine, Anhui Medical College, No. 632 of Furong Road, Shushan District, Hefei, 230601 Anhui, China; ^2^Department of Urology, The First Affiliated Hospital of Anhui Medical University; Institute of Urology, Anhui Medical University; Anhui Province Key Laboratory of Genitourinary Diseases, Anhui Medical University, Hefei 230032, China

## Abstract

**Background:**

Adrenocortical carcinoma (ACC) is a rare and poor prognosis malignancy. Necroptosis is a special type of cell apoptosis, which is regulated in caspase-independent pathways and mainly induced through the activation of receptor-interacting protein kinase 1, receptor-interacting protein kinase 3, and mixed lineage kinase domain-like pseudokinase. A precise predictive tool based on necroptosis is needed to improve the level of diagnosis and treatment.

**Method:**

Four ACC cohorts were enrolled in this study. The Cancer Genome Atlas ACC (TCGA-ACC) cohort was used as the training cohort; three datasets (GSE19750, GSE33371, and GSE49278) from Gene Expression Omnibus (GEO) platform were combined as the GEO testing cohort after removing of batch effect. Forty-nine necroptosis-associated genes were obtained from a prior study and further filtered by least absolute shrinkage and selection operator Cox regression analysis; corresponding coefficients were used to calculate the necroptosis-associated gene score (NAGs). Patients in the TCGA-ACC cohort were equally divided into two groups with the mean value of NAGs. We investigated the associations between NAGs groups and clinicopathological feature distribution and overall survival (OS) in ACC, the molecular mechanisms, and the value of NAGs in therapy prediction. A nomogram risk model was established to quantify risk stratification for ACC patients. Finally, the results were confirmed in the GEO-combined cohort.

**Result:**

Patients in the TCGA-ACC cohort were divided into high and low NAGs groups. The high NAGs group had more fatal cases and advanced stage patients than the low NAGs group (*P* < 0.001, hazard ratio (HR) = 13.97, 95% confidence interval (95% CI): 4.168–46.844; survival rate: low NAGs, 7.69% vs. high NAGs, 61.53%). NAGs were validated to be negatively correlated with OS (*R* = −0.48, *P* < 0.001) and act as an independent factor in ACC with high discriminative efficacy (*P* < 0.001, HR = 11.76, 95% CI: 2.86–48.42). In addition, a high predictive efficacy nomogram risk model was established combining NAGs with tumor stage. Higher mutation rates were observed in the high NAGs group, and the mutation of TP53 may lead to a high T cell infiltration level among the NAGs groups. Patients belonged to the high NAGs are more sensitive to the chemotherapy of cisplatin, gemcitabine, paclitaxel, and etoposide (all *P* < 0.05). Ultimately, the same statistical algorithms were conducted in the GEO-combined cohort, and the crucial role of NAGs prediction value was further validated.

**Conclusion:**

We constructed a necroptosis-associated gene signature, revealed the prognostic value between ACC and it, systematically explored the molecular alterations among patients with different NAGs, and manifested the value of drug sensitivity prediction in ACC.

## 1. Introduction

Adrenocortical carcinoma (ACC) is an ultrarare malignancy originating in the outer layer cortex of the adrenal gland, affecting 0.7-2.0 per million annually and leading to 0.2% of all cancer deaths in the United States [1]. ACC is a hereditary associated syndrome; many underlying genetic alterations have been found, such as TP53, ZNFR3, CTNNB1, PRKAR1A, CCNE1, and TERF2 mutations [2]. In patients diagnosed with ACC, three main scenarios have been reported. First, approximately 40% to 60% of patients showing predominant complaints have hormone excess-related symptoms and signs [3, 4]; hypercortisolism is frequent and often causes plethora, diabetes mellitus, muscle weakness, and osteoporosis. Second, about 30% patients present with nonspecific symptoms due to the growth of tumor, such as abdominal or flank pain, abdominal fullness, or early satiety [3, 5]. Third, the residual roughly 20% of ACCs are incidentally diagnosed by unrelated medical issues [6]. The European Network for the Study of Adrenal Tumors (ENSAT) staging system was recommended at initial diagnosis [7]. Steroid hormone measurements and biochemical exclusion of a pheochromocytoma detection and imaging method are often used to screen ACC [8, 9]. Once diagnosed with ACC, clinicians would treat them with multidisciplinary therapeutic strategies, such as tumor resection [10], adjuvant therapy [11], mitotane [12], and cytotoxic therapy and radiotherapy [13, 14].

Programmed cell death (PCD) is a genetically regulated form of cell death, and apoptosis was historically considered its only form. At present, a special type of necrosis termed necroptosis has also been proven to be a novel form of PCD [15]. Compared to apoptosis, necroptosis is regulated in caspase-independent pathways and is mainly induced by receptor-interacting protein kinase 1 (RIPK1), RIPK3, and mixed lineage kinase domain-like pseudokinase (MLKL). Necroptosis has a morphological resemblance to nonregulated necrosis caused by physical trauma manifesting as organelle swelling, plasma membrane rupture, cell lysis, depletion of energy, and local inflammation [16]. It has been proposed that necroptosis plays a key role in cancer immunity, cancer subtypes, oncogenesis, and metastasis [17]. Accumulated evidence showed that necroptosis is a double-edged sword in cancer. It can prevent tumor development by inducing cancer cell death. However, necroptosis-associated inflammatory reactions may also promote cancer metastasis [18, 19].

In this study, we conducted least absolute shrinkage and selection operator (LASSO) Cox regression using the data from TCGA platform to filter necroptosis-associated genes and calculate the corresponding necroptosis-associated gene score (NAGs). We revealed the correlation between NAGs and overall survival (OS) of ACC and manifested the important value in predicting prognosis and drug sensitivity for patients with ACC. We established a high-performance nomogram risk model for convenient clinical application. Meanwhile, we revealed different molecular mechanisms and gene mutations between the high NAGs and low NAGs groups and validated that immune-related signaling pathways played a pivotal role in ACC development.

## 2. Method

### 2.1. Summary of Cohorts

Four ACC cohorts including transcription profiles and clinical data were downloaded, one was from the Cancer Genome Atlas (TCGA-ACC, https://www.cancer.gov), and three from Gene Expression Omnibus (GEO, http://www.ncbi.nlm.nih.gov/geo/). “TCGAbiolinks” package was used to download mRNA expression profiles of the TCGA-ACC cohort and corresponding clinical information from the Genomic Data Commons (GDC) platform. The original expression data in GSE19750 and GSE33371 cohorts were downloaded and annotated via the corresponding GPL570 platform, while GSE49278 was annotated via the GPL16686 platform. After initial data processing, a total of 167 ACC patients were enrolled for subsequent analysis, including 78 from the TCGA-ACC cohort, 22 from the GSE19750 cohort, 23 from the GSE33371 cohort, and the remaining 44 from the GSE49278 cohort (Table 1). 12 samples from the TCGA-ACC cohort were excluded, due to the lack of clinical information, gene expression profile, or follow-up days less than 1 month. Five normal cases and 21 cases without OS information in GSE19750 were excluded; 10 normal cases, 22 adrenocortical adenoma cases, and 10 cases without OS information in GSE33371 were excluded. All the cases in GSE49278 were enrolled in the study.

### 2.2. Dismissal of Batch Effects

Batch effects are the nonbiological differences between two or more datasets. To eliminate the bias caused by batch effects in this study and make the transcription profiles in the three GEO cohorts more similar, the ComBat algorithms in the “sva” package was used to remove the batch effects between these three GEO-sourced cohorts, and the GEO-combined cohort was used as the testing cohort, while the TCGA-ACC cohort was used as the training cohort in the subsequent analysis (Figures 1(a) and 1(b)).

### 2.3. Construction of the Necroptosis Prognostic Score

A total of 67 necroptosis-associated genes were collected from a recently published article, and after merging with the gene symbols in four enrolled cohorts, 49 necroptosis-associated genes remained for subsequent analysis (Figure 1(c)). A statistical model was generated by LASSO regression analysis performed by the “glmnet” package. We used the LASSO regression to select genes and corresponding coefficients to calculate the NAGs. All the patients in TCGA-ACC cohort and GEO-combined cohort were divided into high and low NAGs groups with the mean NAGs. Based on the TCGA-ACC cohort, the correlation between NAGs and OS and the clinical feature distribution among NAGs groups were further estimated.

### 2.4. Prognostic Prediction with Multivariate Analysis and Nomogram Risk Model

Multivariate analysis was performed to investigate the independent prognostic factors, receiver operating characteristic (ROC) curves were employed, and the area under the curve (AUC) was calculated to test the stability. A nomogram risk model was established by the R package “regplot” to provide a quantitative tool for clinicians for individualized prediction of progression probability. Calibration curves was drawn to assess the model goodness of fit. Decision curve analysis and clinical impact curves quantified the net benefits at different threshold probabilities to determine the clinical usefulness of the nomogram by using the R packages “rms” and “rmda.”

### 2.5. Gene Set Variation Analysis, Immune Infiltration, and Genetic Mutations

We used gene set variation analysis (GSVA) to assess the variations in the pathway activities among patients with high and low NAGs by the “GSVA” R package. The 50 hallmark gene sets were obtained from MSigDB [20, 21]. We used single-sample gene set enrichment analysis (ssGSEA) to investigate the infiltration of 28 immunocytes in tumors and calculate infiltration score of each type of immunocyte for each patient using [22]. A lollipop plot was further drawn to show the correlation between the risk score and infiltration of immunocytes with a *P* value less than 0.05. Anticancer immune response determines the fate of tumor cells and is reflected by the cancer immunity cycle which consists of seven steps: step 1, cancer cell antigens releasing; step 2, cancer antigen presentation; step 3, immune priming and activation; step 4, immunocytes trafficking; step 5, immunocytes infiltration in tumors; step 6, tumor cells recognition by T cells; and step 7, killing of tumor cells [23]. The genetic mutations of ACC patients were also enrolled from the Genomic Data Commons (GDC) by the “TCGAbiolinks” package and further visualized via the “maftools” R package [24].

### 2.6. Precision Therapeutic Strategies

To investigate the therapeutic prediction ability of NAGs, we enrolled gene expression profile from a melanoma cohort which contained 47 cases who received anti-CTLA4 or anti-PD1 therapy and corresponding response information [25]. The gene expression distribution among NAGs groups and potential responders to anti-CTLA4 or anti-PD1 were analyzed using SubMap algorithms via GenePattern platform [26]. For chemotherapy, drug sensitivity and phenotype data from GDSC 2016 (https://www.cancerrxgene.org/) was used to predict the chemotherapeutic response via R package “MOVICS” [27]. Estimated inhibitory concentration (IC50) was set as the index to quantificationally compare the response of each patient treated with a type of chemotherapy drug by ridge regression, and lower IC50 imply increased sensitivity to treatment, and the prediction accuracy was assessed through 10-fold cross-validation [28]. We also downloaded the RNA sequence data from GSE116439 and GSE116444 [29], which contains the data of multiple cell lines treated with or without cisplatin and gemcitabine for 2 hours, 6 hours, and 24 hours, to confirm the predictive value of the necroptosis value for chemotherapy sensitivity.

### 2.7. Statistics

All statistical analyses were performed by R (version: 4.0.2). A Fisher's exact test was used for categorical data and a *t* test or Pearson's correlation analysis was applied for continuous data. A Kaplan-Meier curve was generated by the log rank test to analyze survival rates for patients with different detection methods, and ROC analyses were employed to examine the prediction efficiency of NAGs and performed by the R package “pROC.” A two-tailed *P* value < 0.05 was recognized statistically significant. Hazard ratios (HRs) and 95% confidence intervals (CIs) for OS were estimated via Cox proportional hazard regression. The selected necroptosis-associated prognostic value of NAGs and other features was assessed by the function “ggforest” in the R package “surviminer” and displayed with forest plot. The selected necroptosis-associated genes and clinical features were displayed in heatmap performed by the R package “pheatmap.”

## 3. Results

### 3.1. Establishment of the Prognostic Necroptosis-Associated Gene Signature

Seven necroptosis-associated genes were eventually selected via LASSO and Cox regression analyses under the best optimal lambda value of 0.008, including LEF1, MAPK8, CYLD, TRAF2, DNMT1, PLK1, and GATA3 based on the TCGA-ACC cohort (Figures 2(a) and 2(b)). Each of these genes was proved to be related to the OS of ACC significantly (Fig. S1). NAGs was calculated with the following formula: MAPK8 expression∗0.207 + TRAF2 expression∗0.0506 + DNMT1 expression∗0.181 + PLK1 expression∗0.474 + GATA3 expression∗0.0586 + LEF1 expression∗0.103 + CYLD expression∗(−0.371). We found that NAGs was negatively correlated with the OS of ACC patients, with a *P* value of 8e-06 (Figure 2(c), *R* = −0.48). Seventy-eight patients in the TCGA-ACC cohort were equally divided into low NAGs and high NAGs groups with the median value. In the two new defined groups, different distributions of clinicopathological features between low NAGs and high NAGs groups were observed, including status of survival (*P* = 7.2e − 07) and tumor stage (*P* = 1.7e − 06), but not tumor side (*P* = 0.49) and patient age (*P* = 0.26) or sex (*P* = 1) (Figure 2(d)). ROC analysis manifested a high discriminative efficiency of the necroptosis-associated gene signature, with the AUC values of 0.925 at 1 year, 0.932 at 3 years, and 0.915 at 5 years, respectively (Figure 2(e)). In addition, high and low NAGs groups exhibited clear boundaries (Figure 2(f)). K-M curves demonstrated that patients with low NAGs had significantly longer OS than patients with high NAGs (Figure 2(g), *P* < 0.001, HR = 13.97, 95% CI: 4.168-46.844), and NAGs also exhibited admirable prognostic value in patients with same clinicopathological parameters (Fig. S2).

### 3.2. NAGs Is an Independent Prognostic Predictor of ACC

We enrolled five clinicopathological features and conducted multivariate Cox regression analysis to screen the independent prognostic factors of ACC. The forest plot showed that only NAGs acted as an independent prognostic factor (*P* < 0.001), while age (*P* = 0.5987), gender (*P* = 0.4944), stage (*P* > 0.05), and laterality (*P* = 0.9618) had no statistical significance (Figure 3(a)). The AUC values of different clinicopathological features were calculated to compare their discrimination ability, and the results are shown in Figure 3(b). NAGs with an AUC value of 0.945 (95% CI: 0.887-1.00) and tumor stage with an AUC of 0.831 (95% CI: 0.729-0.933) shows a best predictive efficacy among the five clinicopathological features.

### 3.3. A Nomogram Incorporating the NAGs

Based on the prior results, we established a nomogram risk model combining NAGs and tumor stage to provide a quantitative and precise tool for clinicians to predict progression probability of each patient with ACC (Figure 3(c)). For a given patient, the sum of score for each predictor represented the nomogram score, and a low number of nomogram scores indicated increased progression possibility. Likewise, we verified discrimination of the nomogram risk model via ROC analysis, and the AUC value of 0.967 (95% CI: 0.928-1.00) implied its admirable predictive ability (Figure 3(b)). A *P* value of 0.865 in calibration analysis indicated that the prediction performance of this nomogram might be equivalent to an ideal predictive model (Figure 3(d)). Decision curve analysis (DCA) and the clinical impact curves were performed to demonstrate high clinical net benefit almost over the entire threshold probability of the nomogram model in training cohort (Figures 3(e) and 3(f)).

### 3.4. Different Pathway Activation among NAGs Groups

GSVA revealed the disparities in underlying biological pathways between the high NAGs and low NAGs groups. As the results shown (Figure 4(a)), the high NAGs group has obvious cell cycle changes (including E2F targets and G2M checkpoint pathways), tumor aggression (including MYC targets V1 and MYC targets V2 pathways), and immune suppression (including WNT beta catenin signaling pathways) related pathway activation, while the low NAGs group was with more pathway involving immune activation, including interferon alpha response, interferon gamma response, IL2 STAT5 signaling pathway, inflammatory response, and complement activation pathways [30–32]. Gene mutation is the initial event before tumorigenesis and causes different phenotypes with different manifestations, pathological features, and clinical outcomes in ACC. ACC is a heterogeneity disease with multiple molecular alterations (Fig. S3).Therefore, we further compared the genetic alteration landscape between the two defined groups. The mutation detection rate in the high NAGs group with 74.36% was higher than that in the low NAGs group with 53.85% (Figures 4(b) and 4(c)). The most frequently mutated genes in the high NAGs group included TP53 (31%), CTNNB1 (23%), MUC16 (15%), HMCN1 (15%), MEN1 (15%), and TTN (15%). High MUC16 mutation and CTNNB1 were also observed in the low NAGs group, but their mutation frequencies were different (10% vs. 16% and 8% vs. 23%, respectively). Other gene events, such as COL5A1 (8%), FBN2 (8%), PRKAR1A (8%), and TMEM247 (8%) mutations, were also responsible for the development of low NAGs ACC. Furthermore, ACC with high NAGs has more variable mutation types than ACC with low NAGs. Missense mutation, frameshift deletion, splice site, nonsense mutation, and interframe deletion were all observed in the high NAGs group, while missense mutation, frameshift deletion, splice site, and nonsense mutation were observed in the low NAGs group. Interestingly, NAGs negatively correlated with T cell recruitment (including CD8 T cells and Th1 cells), dendritic cell recruitment, and macrophage and NK cell recruitment but positively correlated with CD4 T cell recruitment, Th22 cell recruitment, and Th2 and Treg cell recruitment in the cancer immunity cycle. Meanwhile, we found that NAGs was negatively correlated with the interferon gamma signature and APM signaling pathways but positively correlated with most signaling pathways shown in the butterfly plot (Figure 4(d)).

### 3.5. NAGs Links with the Response to Anti-PD-1 Immunotherapy

As mentioned above, NAGs was negatively related to immune-related pathway activation. We then employed ssGSEA to investigate the immunocyte infiltration status in the tumor microenvironment (TME). The results showed that multitudinous immunocytes gathered in the TME of ACC with low necroptosis score but rarely in the ACC with high NAGs (Figure 5(a)). Subsequently, we conducted SubMap analysis with an ACC cohort containing both patients who received and did not receive anti-PD-1 or anti-CTLA4 therapy. Patients in the low NAGs group presented a potential better treatment response to anti-PD1 therapy than those in the high NAGs group (Figure 5(b), Bonferroni corrected *P* = 0.018). Furthermore, a checkmate cohort containing four clinical outcomes was enrolled to investigate the relevance of NAGs and different clinical endpoints. Compared to patients with progressive disease (PD), those with stable disease (SD) had obviously higher NAGs (*P* = 0.013) as well as those with partial or complete response (PR/CR) (*P* = 0.4) (Figure 5(c)). Taken together, the evidence proposed above indicated that patients with low NAGs may be more suitable for anti-PD-1 therapy and more likely to obtain clinical benefit.

### 3.6. NAGs Links with the Response to Cisplatin, Gemcitabine, Paclitaxel, and Etoposide Treatment

Based on the data obtained from GDSC 2016, we predicted the sensitivity of four chemotherapeutic agents to patients, including cisplatin, gemcitabine, paclitaxel, and etoposide, and revealed that patients with high NAGs were more suitable for chemotherapy (all *P* < 0.05, Figure 5(d)). A higher IC50 was observed in the low NAGs group in the four classes, suggesting that patients with high NAGs are more sensitive to chemotherapy than those with low NAGs. We analyzed drug-induced changes in NAGs across NCI-60 cell lines after exposure to cisplatin or gemcitabine for 2, 6, and 24 h. NAGs began to decrease after 2 h of exposure to cisplatin (*P* = 0.57), but there was no statistical significance until 6 hours (*P* = 0.028), which continuously decreased within 24 h (*P* = 1.1e − 07) (Figure 5(e)). Similar to the result in cisplatin class, significantly decreased NAGs was observed at 6 h (*P* = 8.3E − 09) and kept declining with 24 h in gemcitabine class (Figure 5(f)).

### 3.7. Validation in GEO-Combined Cohort

After removing the batch effect between the GSE19750, GSE33371, and GSE49278 cohorts, we obtained a GEO-combined cohort with 89 samples. In the GEO-combined cohort, each of the selected necroptosis-related genes were also capable to predict prognosis independently, and the same formula was employed to calculate the NAGs for individual patient (Fig. S4). NAGs was also found negatively associated with OS in ACC (Figure 6(a)). Similarly, 89 samples were further separated into two distinct subgroups with the mean NAGs, high NAGs group with 44 cases, and low NAGs group with 45 cases (Figure 6(d)). We also investigated the clinicopathological distribution between two groups, and the results showed that high NAGs ACC had a higher mortality rate (*P* = 0.00021) and a predisposition of females (*P* = 0.0052). In contrast to the result in TCGA-ACC cohort, there was no staging difference observed among necroptosis-associated gene signature groups (*P* = 0.14), which may be caused by multiple factors, such as the experience of a pathologist, since there was a 13% misdiagnosis rate in ACC [33]. Significant prognostic value was found in the GEO-combined cohort, with 1-year, 3-year and 5-year AUC accuracies of 0.82, 0.826 and 0.858, respectively (Figure 6(C)), and showed a statistically significant OS, with a *P* value less than 0.001 (95% CI: 2.407-8.13) and HR value of 4.43 (Figure 6(e)). For different patient groups with given clinicopathological features in GEO-combined cohort, NAGs was also proved as a good prognostic tool (Fig. S5). According to multivariate analysis, NAGs was reconfirmed as an independent risk factor. Interestingly, tumor stage IV was also validated as the other independent risk factor in the GEO cohort, although there was no statistical significance in the TCGA-ACC cohort (Figure 6(f)). Three parameters, including nomogram, NAGs, and tumor stage, which were found to be high-efficiency prognostic predictors, also demonstrated high predictive ability in the GEO combined cohort, with AUC values of 0.899 (95% CI: 0.837- 0.961), 0.832 (95% CI: 0.745, 0.919), and 0.772 (95% CI: 0.676, 0.867), respectively (Figure 6(g)). Consistently, NAGs negatively correlated with the activation of various immune-related signaling pathways (Figure 7(a)), and more immunocyte infiltration (Figure 7(b)) was observed in the low NAGs group than in the high NAGs group. Patients in the low NAGs group presented a potential better treatment response to anti-PD1 therapy than those in the high NAGs group (Figure 7(c), Bonferroni corrected *P* = 0.011). We also observed a higher sensitivity of cisplatin, gemcitabine, paclitaxel, and etoposide among patients in the high NAGs subgroup, which is similar with the prediction results in TCGA-ACC cohort (all *P* < 0.05, Figure 7(d)).

## 4. Discussion

Adrenal tumors are very common, with an incidence rate of 3%-10% and are mainly diagnosed as small benign nonfunctional adrenocortical adenomas [34]. However, ACC is a rare but aggressive type among adrenal tumors. The overall prognosis of ACC is poor but heterogeneous, with a 5-year survival ranging from 13% to 81%. The challenge faced by clinicians in managing ACC after resection is to select a suitable chemotherapeutic scheme for different patients, while limited parameters can be used for efficacy prediction, and only an ENSAT staging system is available to date. However, survival differences were still reported at a given ENSAT stage in ACC due to genetic heterogeneity [35]. Therefore, it is imperative to uncover the underlying molecular mechanisms in ACC development and provide a complementary method for risk stratification and therapeutic prediction.

The value of molecular markers in distinguishing patients with different risks has been demonstrated in many cancers, such as prostate-specific antigen (PSA) in prostate cancer. Immunohistochemistry of Ki67 in the ACC tumor is a standard to assess the cell proliferation status; several studies already reported the prognostic value of Ki67 in ACC. Beuschlein et al. [36] reported that Ki67 in a powerful prognostic factor to the disease-free survival of ACC patients after surgery, grade 1 ACC with the positive staining of Ki67 less than 10%, grade 2 with positive area between 10 and19%, and Ki67-positive area higher than 20% links with grade 3 ACC tumors. Duregon et al. proved Ki-67 to be the best prognostic indicator of overall survival, being superior to the mitotic index [37]. However, Libé et al. [38] revealed that the prognostic value of Ki67 did not show a good performance in the OS prediction of ACC patients with advanced stage III and IV tumors. Martins-Filho et al. [39] also demonstrated that the prognostic value of Ki67-positive rate is not consistent among adults and pediatrics; in adults, Ki67 ≥ 10% showed the highest HR for recurrence, and this value raised to ≥15% in pediatric ACC tumors.

Many cell death mechanisms have been revealed to date, and necroptosis is a novel form of PCD that induces cell death via a caspase-independent pathway and an alternative method for apoptosis. Walz et al. [40] reported that the morphological feature of confluent necrosis in ACC is universal, while the benign adrenocortical adenomas (ACN) completely lack this kind of highly reproducible feature; what is more, the Ki67 levels above 10% were found in more than 96.8% ACC samples and never in ACNs. Pearlstein et al. [41] reported the similar results; necrosis was more frequent in ACCs (93.3%; 14 of 15) compared with benign ACNs (8.7%; 2 of 23). Necrosis is morphologically characterized by rounding of the cell, cytoplasmic swelling, presence of dilated organelles, and absence of chromatin condensation, while necrotic cell death is carried out by complex signal transduction pathways and execution mechanisms [42, 43]. The results from prior studies showed that some necroptosis-associated genes, such as RIPK1, RIPK3, and MLKL, can be used as prognostic markers in tumors. For instance, Feng et al. found that low expression of RIPK3 was related to a short OS and disease-free survival in colorectal cancer [44]. McCormick et al. demonstrated that low expression of RIPK1 promoted the progression of neck squamous carcinoma [45]. In this study, we conducted a necroptosis-associated gene signature for ACC using LASSO Cox regression analyses based on the TCGA-ACC cohort. We revealed that the necroptosis-associated gene signature was negatively correlated with OS in ACC. Further survival analysis proved significantly different OS among necroptosis-associated gene signature groups. Multivariate Cox regression analysis validated that the signature could act as an independent risk factor in ACC.

To screen clinicopathological parameters with high predictive value, ROC analysis was performed to calculate the corresponding AUC, and tumor stage was eventually enrolled. Combining NAGs with tumor stage, we established a nomogram risk model to quantify the probabilities of tumor progression. Compared to the ENSAT staging system, this novel nomogram model included extra molecular parameters, showed higher clinical net benefit, and presented excellent accuracy of prediction. We believe that it could be a novel diagnostic complement tool for orthodox management of ACC.

An up to 40%-70% recurrence rate has been reported in ACC even after surgical resection, which is higher than most malignancies. Adjuvant therapy is often used as a means of preventing postoperative recurrence. A randomized controlled phase 3 clinical trial proposed that combination adjuvant therapy with etoposide, doxorubicin, cisplatin, and mitotane is the frontline treatment in advanced ACC, but progression-free survival (PFS) and OS, with 5.6 months and 14.8 months, respectively, were still short [46]. Gemcitabine is a salvage regimen once preliminary chemotherapy fails, and the disease control rate is as low as 30% [47]. Meanwhile, there are no ideal tools that can be used to select suitable patients for chemotherapy. We revealed that NAGs can predict the efficacy of etoposide, cisplatin, gemcitabine, and paclitaxel in the treatment of ACC. In addition, we observed that NAGs declined after receiving gemcitabine treatment or cisplatin treatment in NCI-60 cell lines. Since NAGs is negatively associated with the OS of ACC, the significance of chemotherapy in improving prognosis has been reconfirmed. Although patients with low NAGs are not suitable for immunotherapy, chemotherapy can bring new hope to these patients.

At present, limited treatment options are available for advanced ACC [7]. Immunotherapy provides new options for altering the routine strategies of advanced ACC, and the value of immune checkpoint inhibitor (ICI) therapy has been proposed in many studies. However, the results of a multicenter study of four ICI drugs hint at a poor overall response rate and progression-free survival in treating ACC [48]. Several pathway alterations and molecular alterations may be responsible for ICI therapy resistance, and further immunological markers of response might solve this dilemma. According to a published review, immunocyte infiltration status is the main influencing factor affecting the effectiveness of immunotherapy [49]. High immunocyte infiltration, especially T cells, is generally related to a high response. In ACC, WNT-*β* catenin pathway activation was related to the decreased recruitment of the specific lineage basic leucine zipper transcription factor ATF-like 3 lineage (BATF3) of dendritic cells, which is associated with the production of chemokines such as CXCL9 and CXCL10, leading to the downregulation of T cell infiltration. In addition, upregulation of TP53 inactivating mutations leads to the lack of production of pivotal chemokines in T cells and natural killer recruitment, which contribute to the exclusion of T cytotoxicity from the tumor microenvironment and reduced activation of cytotoxicity-related chemokines. In our study, WNT pathway activation and a high TP53 mutation rate were observed in ACC with high NS, and on the other hand, ACC with low NAGs had substantive immune-related pathways and immunocyte recruiting pathway activation. All these results indicated higher immunocyte infiltration and a good response in low NAGs group than in the high NAGs group. As expected, further ssGSEA and SubMap analyses validated them, and patients with PD tended to have a higher NAGs than those with SD, PR, or CR. The evidence mentioned above indicates that the necroptosis-associated gene signature may be a promising predictor for ICI therapy. We constructed a necroptosis-associated gene signature associated with the prognosis of ACC, revealed molecular mechanisms of high-risk ACC, and found the value of drug sensitivity prediction. We established a nomogram risk model to quantify the risk stratification of ACC and wish to provide a high-efficacy predictive tool for clinicians. But there are still some limitations. For instance, more expression products of the seven genes that can be detected by a cheap means are needed to concern, and the sample size is small as there are only 167 cased enrolled in our study. In conclusion, we generated a novel multigene predictor which can make a contribution to the OS prediction of ACC.

## Figures and Tables

**Figure 1:** Data exhibition and processing of four cohorts. (a). Row principal coordinates analysis (PCA) for the combined expression profile from the GSE19750, GSE33371, and GSE49278 cohorts. (b) PCA for the combined expression profile from the three cohorts after removing batch effects. (c) Heatmap showed the distributions of clinical information and 49 necroptosis-associated genes in four cohorts.

**Figure 2:** LASSO Cox regression selected necroptosis-associated genes with the best optimal lambda value, the association between NAGs and clinical features, and the survival analysis among NAGs groups. (a) The coefficients of 49 necroptosis-associated genes. (b) The seven necroptosis-associated genes selected with the best optimal lambda value, including LEF1, MAPK8, CYLD, TRAF2, DNMT1, PLK1, and GATA3. (c) The negative correlation between NAGs and OS in ACC. (d) Distribution of clinicopathological, status of survival, and tumor stage among NAGs groups. (e) Predictive accuracy of necroptosis-related gene signature at 1 year, 3 years, and 5 years, and the accuracy was equal to the corresponding AUC value. (f) Two distinct subgroups divided by the mean NAGs. (g) Different survival probabilities between the two defined subgroups are showed in K-M curves.

**Figure 3:** Multivariate Cox regression was performed to validate independent prognostic factors in ACC, and a nomogram model was established to predict progression risk for each patient. (a) Forest plot of corresponding multivariate HR for six algorithms, including age, gender, stage, laterality, and NAGs. Tumor stages assessed at stage I, stage II, stage III, stage IV, and unknown because of the pivotal effects on prognosis. Lines that do not cross the dashed line are considered as independent prognostic factors. (b) Discriminative power of four clinicopathological features as well as the nomogram and NAGs; the accuracy was equal to corresponding AUC value, and the value more than 0.75 represents high stability. (c) Establishment of a nomogram combining tumor stage and NAGs. For a given patient, find patient's tumor stage on stage axis, find patient's NAGs on NAGs axis, each time draw straight line upward toward points axis, total points were the sum of each predictor point, find the total point on total point on total point axis, draw straight line to the bottom 3-year progression probability and 5-year progression probability axis, and the points in progression line represented the progression probability. (d) Calibration plot for the nomogram. The dashed line represents the ideal nomogram, the solid line represents our nomogram, and a *P* value of 0.865 indicates that our nomogram is very close to the ideal nomogram. (e) DCA showed that our nomogram had the greatest net benefit among the four policies. (f) The clinical impact curve for the predictive value of the nomogram model, the orange solid line represents the predictive number of patients with high risk, and the black dashed line represents the actual number of patients with high risk.

**Figure 4:** Pathway activation and gene mutations among NAG groups were revealed. (a) Different metabolic pathways between high and low NAGs groups; the significant activation pathways were marked with purple and green. (b) Different gene alterations between the two groups, and different spectral color represent different types of genetic mutation. (c) Correlations between NAGs and the steps of the cancer immunity cycle and correlations between NAGs and the enrichment scores of immunotherapy-predicted pathways. The dashed lines represent a negative correlation, and the solid lines represent a positive correlation.

**Figure 5:** The immunocyte infiltration landscape of ACC was revealed by ssGSEA, and a necroptosis-associated gene signature was validated as a predictor for both immunotherapy and chemotherapy in ACC. (a) Immunocyte infiltration landscape for each patient depiction via a heatmap. (b) Response prediction of immunotherapy via SubMap analysis with an ACC cohort containing both patients who received and did not receive anti-PD1 or anti-CTLA4 therapy. (c) Comparison of NAGs among patients with CP/RP, PD, and SD in a checkmate cohort. (d) Comparison of chemotherapy response between high and low NAGs groups. The IC50 was employed as the evaluation indicator, and a higher IC50 represented lower drug sensitivity. (e) Drug-induced change in NAGs across NCI-60 cell lines after exposure to cisplatin for 2, 6, and 24 h. (f) Drug-induced change in NAGs across NCI-60 cell lines after exposure to gemcitabine for 2, 6, and 24 h.

**Figure 6:** Clinical relevance and survival analyses in the GEO combined cohort. (a) Correlations between NAGs and OS. (b) Comparisons of clinicopathological feature distributions between the high and low NAGs groups. (c). Discriminative accuracy validation in GEO combined cohort; ROC analysis was conducted to calculate the AUC value at 1 year, 3 years, and 5 year, respectively. (d). High and low NAGs patients in GEO combined cohort. (e) Comparisons of OS between patients with high NAGs and low NAGs, the results were depicted via K-M curves. (f) Multivariate Cox regression analysis.

**Figure 7:** Pathway enrichment analysis and therapeutic response to immunotherapy and chemotherapy in ACC based on the GEO combined cohort. (a) Enrichment analysis of metabolic pathways in the low NAGs group and high NAGs group via GSVA algorithms and comparison of enrichment scores. (b) Tumor immunocyte infiltration landscape of patients in GEO combined cohort. (c) Assessment of therapeutic response to anti-CTLA4 and anti-PD-1 in ACC D. Comparison of response to four chemotherapy agents, including cisplatin, gemcitabine, paclitaxel, and etoposide.

**Table 1:** Basic clinical features of cohorts enrolled in the current study.

	TCGA_ACC (*n* = 78)	GSE19750 (*n* = 22)	GSE33371 (*n* = 23)	GSE49278 (*n* = 44)	Total (*n* = 167)
Gender					
Female	47 (60.3%)	11 (50.0%)	16 (69.6%)	36 (81.8%)	110 (65.9%)
Male	31 (39.7%)	11 (50.0%)	7 (30.4%)	8 (18.2%)	57 (34.1%)
Age					
Mean (SD)	46.7 (15.9)	52.5 (14)	43 (16.8)	45.1 (17.2)	46.5 (16.2)
Median [min, max]	49.5 [14,77]	54.6 [23.3,72.1]	45 [10,77]	43.5 [15,81]	48 [10,81]
Stage					
Stage I	9 (11.5%)	1 (4.5%)	2 (8.7%)	4 (9.1%)	16 (9.6%)
Stage II	37 (47.4%)	7 (31.8%)	10 (43.5%)	24 (54.5%)	78 (46.7%)
Stage III	16 (20.5%)	1 (4.5%)	3 (13.0%)	2 (4.5%)	22 (13.2%)
Stage IV	14 (17.9%)	4 (18.2%)	8 (34.8%)	13 (29.5%)	39 (23.4%)
Unknown	2 (2.6%)	9 (40.9%)		1 (2.3%)	12 (7.2%)
Side					
Left	44 (56.4%)		10 (43.5%)	23 (52.3%)	77 (46.1%)
Right	34 (43.6%)		10 (43.5%)	21 (47.7%)	65 (38.9%)
Unknown		22 (100.0%)	3 (13.0%)		25 (15.0%)

## Data Availability

The data used to support the findings of this study are available from the corresponding author upon request.

## Supplementary Materials

Supplementary Materials Figure S1: K-M plot showing the prognostic value of seven selected genes in TCGA-ACC cohort. Figure S2: K-M plot showing the prognostic value of NAGs among different clinical subgroups in TCGA-ACC cohort. Figure S3: summary of the mutations in ACC patients from TCGA-ACC cohort. Figure S4: K-M plot showing the prognostic value of seven selected genes in combined GEO cohort. Figure S5: K-M plot showing the prognostic value of NAGs among different clinical subgroups in combined GEO cohort.
